The article "Comparative Efficacy of Semaglutide Versus Liraglutide or Efinopegdutide on Weight Loss in Obese Patients: A Systematic Review and Meta-Analysis" was published in 2024. Journal: Cureus.

# Comparative Efficacy of Semaglutide Versus Liraglutide or Efinopegdutide on Weight Loss in Obese Patients: A Systematic Review and Meta-Analysis

**DOI:** 10.7759/cureus.75304

**Published:** 2024-12-07

**Authors:** Jimmy Wen, Christiane How-Volkman, Alina Truong, Denise Nadora, Ethan M Bernstein, Muzammil Akhtar, Jose Puglisi, Eldo Frezza

**Affiliations:** 1 Physical Medicine and Rehabilitation, California Northstate University College of Medicine, Elk Grove, USA; 2 College of Medicine, California Northstate University College of Medicine, Elk Grove, USA; 3 Cardiology, California Northstate University College of Medicine, Elk Grove, USA; 4 Neurology, California Northstate University College of Medicine, Elk Grove, USA; 5 Orthopedic Surgery, California Northstate University College of Medicine, Elk Grove, USA; 6 Surgery, California Northstate University College of Medicine, Elk Grove, USA; 7 Biostatistics, California Northstate University College of Medicine, Elk Grove, USA

**Keywords:** efinopegdutide, glp-1 agonist, liraglutide, obesity and overweight, semaglutide, weight loss

## Abstract

Glucagon-like peptide-1 agonists (GLP-1 RAs) have produced substantial weight loss effects in type 2 diabetes mellitus (T2DM) cohorts, but these effects have not been thoroughly studied in patients with obesity and without diabetes. This review aimed to analyze direct comparative studies for semaglutide versus other GLP-1 RA (liraglutide and efinopegdutide) in facilitating weight loss and evaluating adverse events in patients with obesity. A systematic search following the guidelines established by the Preferred Reporting Items for Systematic Reviews and Meta-Analyses (PRISMA) was performed in PubMed, Embase, and Cochrane Library for direct comparative studies comparing semaglutide with other GLP-1 RA on weight loss in patients with obesity. A narrative synthesis and meta-analysis were performed to analyze the differences in weight loss between cohorts.

A meta-analysis found that semaglutide produced a greater effect on mean weight loss compared to liraglutide, but did not produce a significant difference compared to efinopegdutide. Semaglutide, liraglutide, and efinopegdutide were well-tolerated and were associated with primarily minimal to moderate severity adverse effects, most of which were gastrointestinal. Future studies should continue to focus on conducting direct comparisons between GLP-1 RAs and emerging multi-receptor GLP-1 RAs, such as efinopegdutide, tirzepatide, and retratrutide, to determine clinical efficacy, long-term safety, and identifying the most effective regimens for clinical practice.

## Introduction and background

Obesity continues to emerge as an alarming global health epidemic, posing long-term challenges for healthcare systems as well as patients’ daily routines and comorbidities such as cardiovascular disease, diabetes, and several cancers including but not limited to breast, colorectal, kidney, pancreatic, and liver [1,2]. Patients with obesity were previously limited to a handful of Food and Drug Administration (FDA)-approved drugs (e.g., orlistat, phentermine-topiramate, bupropion-naltrexone) to manage obesity, with varying efficacy [1]. Recently, the ability of glucagon-like peptide-1 receptor agonists (GLP-1 RAs) to produce weight loss has been attributed to their effects on increasing insulin secretion, decreasing glucagon levels, suppressing appetite, and enhancing satiety. Additionally, these weight loss effects are augmented by delayed gastric emptying and stimulation of central receptors that control appetite suppression and energy expenditure [3]. With an evidence-based understanding of the efficacy and safety profiles of GLP-1 RAs for obesity, research can aid healthcare systems in allocating resources and personalizing treatment.

The article "Comparative Efficacy of Semaglutide Versus Liraglutide or Efinopegdutide on Weight Loss in Obese Patients: A Systematic Review and Meta-Analysis" was published in 2024. Journal: Cureus.

Liraglutide 3.0 mg daily subcutaneous (SQ) injection was the first FDA-approved GLP-1 agonist approved for weight loss in patients with obesity and semaglutide 2.4 mg weekly SQ injection followed shortly after [4]. While GLP-1 RAs are efficient in promoting weight loss in diabetic patients, current points of interest include understanding the effect of GLP-1 RAs in individuals with obesity, as few studies encompass direct comparisons of GLP-1 RAs for this purpose.

This systematic review aimed to evaluate existing comparative studies regarding the impact of semaglutide compared to another GLP-1 RA (liraglutide and efinopegdutide) in facilitating weight reduction and safety profile in patients with obesity [5]. Comparative studies rather than indirect comparisons/network meta-analyses reduce the bias inherent in differing patient demographics and provide a more accurate reporting of weight loss and complications. The goal of this comprehensive analysis is to provide insights for clinicians and patients when selecting a GLP-1 RA, as well as to identify gaps in the current literature that can be explored further to optimize patient outcomes and quality of life.

## Review

Methods

Search Strategy

This systematic review followed the guidelines indicated in Preferred Reporting Items for Systematic Reviews and Meta-Analyses (PRISMA). All authors participated in identifying the articles included in this study. The search was conducted in the following three databases on 15 November 2023: Cochrane Library, Embase, and PubMed. All three databases were searched using the following search strategy: Semaglutide AND (exenatide OR liraglutide OR albiglutide OR dulaglutide OR lixisenatide OR tirzepatide OR GLP-1 agonist OR glucagon-like peptide-1 agonist) AND (weight loss). No specific limits were placed on our search strategy to ensure that no articles related to any GLP-1 agonists were missed.

The article "Comparative Efficacy of Semaglutide Versus Liraglutide or Efinopegdutide on Weight Loss in Obese Patients: A Systematic Review and Meta-Analysis" was published in 2024. Journal: Cureus.

Article Selection Process

A patient, intervention, comparison, and outcome (PICO) method was used. In our study, the patient population included patients with obesity only. The intervention includes patients who received either semaglutide or any other GLP-1 agonist. The outcomes of this study included weight loss and side effects that occurred during the administration of the treatment. Exclusion criteria included non-human studies, case reports, reviews, cadaveric studies, expert opinions, conferences, abstracts, and articles not in English. Each article included in the study underwent title and abstract screening by two reviewers. In cases where their decisions were not in agreement, the articles underwent additional review until a consensus was reached to determine their inclusion. Articles that met the initial inclusion criteria underwent a more thorough full-text review. Similarly, to be added to the systematic review, each article required unanimous decisions by two reviewers. This protocol is registered in PROSPERO under the number CRD42023481900.

Risk of Bias Assessment

Two independent authors scored each based on their study quality and to determine the risk of bias using the Methodologic Index for Nonrandomized Studies (MINORS) criteria [6]. The MINORS items are allocated scores of 0 (if not reported), 1 (if reported but inadequate), or 2 (if reported and adequate). In the case of comparative studies, the maximum ideal score is 24. Each author independently reviewed and scored the articles, and their assessments were subsequently compared. Any disparities in the scores were addressed by a re-evaluation of the articles until a consensus was achieved. A study is considered a low risk of bias classification if it receives a MINORS criteria score of 1 or 2 in 11 or more categories. In the case of receiving a score of 1 or 2 in nine or 10 categories, it would be categorized as a moderate risk of bias. Lastly, if a study scores 1 or 2 out of 8 or fewer categories, it is designated as having a high risk of bias. The Cochrane risk of bias tool was also utilized to determine study quality for RCT studies [7]. The tool analyzes sequence generation, allocation concealment, blinding of participants and personnel, blinding of outcome assessment, incomplete outcome data, selective outcome reporting, and other sources of bias as “high risk,” “low risk,” or ”unclear” risk of bias. Any discrepancies were resolved via rigorous re-review until a consensus was reached.

The article "Comparative Efficacy of Semaglutide Versus Liraglutide or Efinopegdutide on Weight Loss in Obese Patients: A Systematic Review and Meta-Analysis" was published in 2024. Journal: Cureus.

Data Extraction and Analysis

The variables that were included in this systematic review include title, author, year of publication, obese status, study design, study period, sample size, gender, mean age, pre-existing medical conditions, dosage, type of intervention given to the patient, mean follow-up time, pre-intervention baseline values, post-intervention values, and key complications of the treatment intervention. If applicable and available, pertinent descriptive statistics (mean, median, standard deviations, ranges) are incorporated. The program SPSS version 29 (Armonk, NY: IBM Corp.) was used to perform a meta-analysis with a random-effect model to compare mean weight loss between GLP-1 RAs. A forest plot was created using GraphPad Prism version 10 (Boston, MA: Dotmatics).

The initial search yielded 2148 articles from PubMed, Embase, and Cochrane Library. The articles were screened for duplicates and subsequently underwent title/abstract screening, and full-text review, which yielded five studies to be included in this systematic review. The screening process is further detailed in Figure 1.

**Figure 1:** PRISMA flow diagram depicting article selection process. PRISMA: Preferred Reporting Items for Systematic Reviews and Meta-Analyses

Demographic Data

Across the five studies, there were 1697 patients, of which 1595 patients completed the study at the final follow-up [4,5,8-10]. The mean age was 50.13 years, with the mean ages ranging from 47.0 to 55.15 years (Table 1).

**Table 1:** Patient demographics of the included studies. *The reported median and interquartile range were used to approximate the weighted average age, with the mean age calculated using the median values.

Studies	Number of patients enrolled	Number of patients who completed the study	Sex (female, male)	Mean age in years (SD)
Jensen et al. (2023) [5]	50	50	41, 9	50 (44.3, 57.8)*
Murvelashvili et al. (2023) [8]	207	207	186, 21	55.15 (10.64)
O'Neil et al. (2018) [4]	957	891	619, 338	47 (12)
Rubino et al. (2022) [10]	338	312	265, 73	49 (13)
Romero-Gómez et al. (2023) [9]	145	135	65, 80	49.5

Study Characteristics

There was a total of three randomized controlled trials (RCTs) and two retrospective cohort studies that met inclusion criteria. Four studies included the comparison of semaglutide and liraglutide, while one included semaglutide versus the comparator of efinopegdutide. Of the studies that studied the differences between semaglutide and liraglutide, two included the analysis of a 1.0 mg weekly dosage of semaglutide versus a 3.0 mg daily dosage of liraglutide. The remaining two studies differed as one compared varying semaglutide escalation regimens to 3.0 mg liraglutide, and the second included a 2.4 mg weekly semaglutide dosage. The mean follow-up period was 44 weeks, ranging from 24 to 68 weeks across studies (Table 2).

The article "Comparative Efficacy of Semaglutide Versus Liraglutide or Efinopegdutide on Weight Loss in Obese Patients: A Systematic Review and Meta-Analysis" was published in 2024. Journal: Cureus.

**Table 2:** Study characteristics of the included studies.

Studies	Number of patients assigned to semaglutide	Semaglutide intervention	Number of patients assigned to comparator	Comparator intervention	Number of patients assigned to placebo	Mean follow-up (months)
Jensen et al. (2023) [5]	21	1.0 mg semaglutide weekly subcutaneous injection (n=20), 14 mg semaglutide daily oral intake (n=1)	29	3.0 mg daily subcutaneous injection liraglutide (n=28), 1.8 daily subcutaneous injection liraglutide (n=1)	0	6
Murvelashvili et al. (2023) [8]	115	1.0 mg semaglutide once weekly	92	3.0 mg daily liraglutide	0	12
O'Neil et al. (2018) [4]	718	Semaglutide: 0.05 mg/day, 0.1 mg/day, 0.2 mg/day, 0.3 mg/day, 0.4 mg/day, 0.3 mg Fast 2 weekly dose escalation (FE)/day, 0.4 mg FE/day	103	3.0 mg daily liraglutide	136	12
Rubino et al. (2022) [10]	126, 86.2% completed	2.4 mg semaglutide once weekly	127, 95.7% completed	3.0 mg daily liraglutide	85	17
Romero-Gómez et al. (2023) [9]	73, 71% completed	1.0 mg semaglutide once weekly	72, 64% completed	10.0 mg once weekly dosage of efinopegdutide	0	6

For study quality and risk of bias assessment, the MINORS and Cochrane risk of bias tools were utilized as this study included both RCTs and non-RCTs. The included studies had MINORS scores ranging from 13 to 22. Overall risk of bias was high in one study, medium in two studies, and low in two studies. The MINORS score is summarized in Table 3.

**Table 3:** Methodological quality and risk of bias.

Studies	Clearly stated aim	Inclusion of consecutive patients	Prospective data collection	Endpoints appropriate to study aim	Unbiased assessment of study endpoint	Follow-up period appropriate to study aim	Loss to follow-up less than 5%	Prospective calculation of study size	Adequate control group	Contemporary groups	Baseline equivalence of groups	Adequate statistical analyses	Total score
Jensen et al. (2023) [5]	2	2	2	2	0	1	0	0	1	0	1	2	13/24
Murvelashvili et al. (2023) [8]	2	2	2	2	0	2	2	0	1	0	1	2	16/24
O'Neil et al. (2018) [4]	2	2	2	2	2	2	0	2	2	2	2	2	22/24
Romero-Gómez et al. (2023) [9]	2	2	2	2	1	1	2	0	1	2	2	2	19/24
Rubino et al. (2022) [10]	2	2	2	2	1	2	0	2	2	2	2	2	21/24

For the Cochrane risk of bias, there was a low risk of bias for incomplete outcome data and selective outcome reporting. Sequence generation and allocation concealment were low in two studies, but there was an unclear risk of bias in one study. The blinding of participants, personnel, and outcome assessors was either at high risk or unclear risk of bias. Finally, for other sources of bias, there were two high risks of bias and one low risk of bias. The risk of bias for the three RCTs, assessed using the Cochrane risk of bias tool is summarized in Table 4.

The article "Comparative Efficacy of Semaglutide Versus Liraglutide or Efinopegdutide on Weight Loss in Obese Patients: A Systematic Review and Meta-Analysis" was published in 2024. Journal: Cureus.

**Table 4:** Cochrane risk of bias tool.

Studies	Sequence generation	Allocation concealment	Blinding of participants and personnel	Blinding of outcome assessors	Incomplete outcome data	Selective outcome reporting	Other sources of bias
O'Neil et al. (2018) [4]	Low	Low	High	Unsure	Low	Low	High
Romero-Gómez et al. (2023) [9]	Unsure	Unsure	Unsure	Unsure	Low	Low	Low
Rubino et al. (2022) [10]	Low	Low	High	Unsure	Low	Low	High

Weight Loss

Weight loss was assessed by calculating the percentage change in weight after GLP-1 RA intervention. Four studies compared semaglutide against liraglutide in affecting weight loss, and three demonstrated semaglutide’s significant effect in facilitating weight reduction. Meta-analysis of all four studies comparing semaglutide and liraglutide revealed an overall significantly greater effect on mean weight loss with semaglutide compared to liraglutide (SMD: -6.39, 95% CI: -9.40, -3.38) (Figure 2). Meanwhile, semaglutide, compared to efinopegdutide, did not produce a significant difference in weight loss, with reductions of 7.51% and 8.58%, respectively (Table 5).

**Figure 2:** Effect of semaglutide versus liraglutide on body weight.

**Table 5:** Effect of semaglutide on body weight compared to liraglutide and efinopegdutide. SD: standard deviation; NR: not reported

Studies	Pre-semaglutide intervention, kg	Post-semaglutide intervention, kg	Weight change percentage	Pre-comparator intervention	Post-comparator intervention	Weight change percentage
Jensen et al. (2023) [5]	NR	NR	-9.80	NR	NR	-7.30
Romero-Gómez et al. (2023) [9]	94.5 (18.9)	87.4 (19)	-7.51	100.2	91.6 (19.5)	-8.58
Murvelashvili et al. (2023) [8]	110.7 (24.50)	96.4	-12.92	114.4 (27.6)	104.4	-8.77
O'Neil et al. (2018) [4]	111.3 (23.2)	104.6	-6	108.7 (21.9)	100.23	-7.79
	111.3 (21.5)	101.7	-8.6			
	114.5 (24.5)	101.2	-11.6			
	111.5 (23)	99.0	-11.2			
	113.2 (26.4)	97.6	-13.8			
	108.1 (22.1)	95.8	-11.4			
	109.6 (21.3)	91.2	-16.8			
Rubino et al. (2022) [10]	102.5 (25.3)	87.2	-15.80	103.7 (22.5)	96.9	-6.40

Factors Associated With Weight Loss

Jensen et al. included a population that experienced weight regain following bariatric surgery. It was reported that treatment with semaglutide was associated with a significantly higher reduction in weight at 9.8% compared to a 7.3% reduction in the liraglutide cohort (p<0.05). There was a pattern of increased weight loss for those patients who began GLP-1 RA treatment at or after 72 months post-bariatric surgery compared to those who began the GLP-1 RA intervention prior to 72 months, though this difference was not statistically significant. Further analysis of potential factors was conducted including factors such as baseline characteristics, diagnosis of type 2 diabetes, sex, age, the presence of anatomical cause for weight regain, and self-payer status. However, no significant findings have been produced on the effect of GLP-1 RAs on weight [5].

The article "Comparative Efficacy of Semaglutide Versus Liraglutide or Efinopegdutide on Weight Loss in Obese Patients: A Systematic Review and Meta-Analysis" was published in 2024. Journal: Cureus.

Furthermore, Murvelashvili et al. also investigated the effect of GLP-1 RAs on patients with weight regain following post-metabolic and bariatric surgery (MBS). Murvelashvili et al. reported that the MBS procedure type of vertical sleeve gastrectomy demonstrated a correlation between the pre-MBS and post-MBS weight as well as weight loss after 12 months of GLP-1 RA treatment; however, there was no significant correlation between those who underwent adjustable gastric banding and Roux-en-Y gastric bypass. Interestingly, there is a positive correlation between post-MBS weight loss and weight loss following GLP-1 RA treatment at the one-year follow-up period, meaning weight loss results following MBS may be further enhanced via GLP-1 RAs (r=0.206, p=0.035) [8].

The study by O’Neil et al. differed from many other studies as it included many dosing regimens and escalation schedules. Patients in the active interventions were categorized into groups receiving 0.05 mg, 0.1 mg, 0.3 mg, or 0.4 mg semaglutide or 3.0 mg liraglutide. Additionally, across groups, semaglutide was started at a dose of 0.05 mg and increased every four weeks, depending on the cohort. Additional groups were prescribed 0.3 mg and 0.4 mg semaglutide and were assigned an exploratory escalation schedule, defined as increasing dosages every two weeks instead of every four weeks. O’Neil reported that semaglutide administration demonstrated a dose-dependent relationship for weight loss. Additionally, semaglutide doses of 0.2 mg or higher demonstrated significant weight loss that towered those in the 3.0 mg liraglutide cohort after one year of treatment [4].

Rubino et al. discussed how the approved prescribing information and dosing regimen of liraglutide could lead those who have AEs to be more prone to discontinue the trial. For example, the process of restarting the dose of liraglutide results in less time for liraglutide to demonstrate its optimal weight loss result, possibly owing to its decreased weight loss profile [10].

Romero-Gómez et al.'s primary endpoint was to determine the effect of GLP-1 RAs on liver fat content in non-alcoholic fatty liver disease (NAFLD). The results demonstrated that efinopegdutide achieved larger weight loss and relative reductions in liver fat content (LFC) compared to semaglutide. Additionally, if there were higher rates of weight loss, there were associated decreases in LFC [9].

The article "Comparative Efficacy of Semaglutide Versus Liraglutide or Efinopegdutide on Weight Loss in Obese Patients: A Systematic Review and Meta-Analysis" was published in 2024. Journal: Cureus.

Adverse Events

This study focused on total AEs, including common adverse events (AEs) such as gastrointestinal events and discontinuations. AEs affected between 36% and 96.1% of the study population. Gastrointestinal events ranged from 38% to 84.1% across studies. There was a wider range of discontinuations due to AEs across cohorts taking liraglutide and efinopegdutide, 4.2-12.6%, compared to those patients assigned to semaglutide therapy, 3.2-8.9%. Jensen et al. included AEs across the total study population and not between comparator cohorts, while Murvelashvili et al. did not report AEs. Table 6 details these AEs and their occurrence in the study populations [5,8].

**Table 6:** Common adverse events with an emphasis on gastrointestinal events. AE: adverse events; NR: not reported

Adverse events	Semaglutide			Active comparator			Total		
	O'Neil et al. (2018) [4]	Rubino et al. (2022) [10]	Romero-Gómez et al. (2023) [9]	O'Neil et al. (2018) [4]	Rubino et al. (2022) [10]	Romero-Gómez et al. (2023) [9]	Jensen et al. (2023) [5]	O'Neil et al. (2018) [4]	Rubino et al. (2022) [10]
Total adverse events	NR	95.20%	72.60%	NR	96.10%	88.90%	36%	NR	NR
Gastrointestinal	73.3%	84.10%	NR	56.5%	82.70%	NR	NR	NR	38%
Nausea	44.1%	NR	31.50%	31.5%	NR	27.80%	22%	18%	NR
Obstipation/constipation	21.1%		5.50%	13.5%		16.70%	10%	4%	
Vomiting	17.3%		15.10%	7.5%		16.70%	2%	4%	
Flatulence	NR		1.40%	NR		5.60%	2%	NR	
Diarrhea	27%		17.80%	20%		16.70%	2%	12%	
Headache	12.6%		6.80%	13%		6.90%	2%	11%	
Discontinuations due to AE	8.9%	3.20%	0.00%	8.7%	12.60%	5.6%, drug-related AE: 4.20%	NR	8%	NR

Discussion

This systematic review analyzed five studies (three RCTs/two non-RCTs) evaluating weight loss outcomes in patients with obesity treated with semaglutide compared to liraglutide and efinopegdutide. Four studies evaluated semaglutide versus liraglutide and one analyzed semaglutide versus a GLP-1/glucagon receptor co-agonist efinopegdutide. Semaglutide, liraglutide, and efinopegdutide were well tolerated and associated with significant weight loss compared to placebo.

Weight Loss

A recent 2022 systematic review and meta-analysis of 12 RCTs evaluating liraglutide’s weight loss effect in patients with obesity found a mean weight and body mass index (BMI) loss of 3.35 kg and 1.45 kg/m^2^, respectively [11]. In Jensen et al.’s study, after six months of semaglutide or liraglutide treatment, there was a reduction of 2.9 kg/m^2^ observed (3.9 kg/m^2^ for semaglutide and 2.5 kg/m^2^ for liraglutide) [5]. O’Neil et al. found a dose-dependent decrease in BMI with escalating semaglutide doses (0.05-0.4 mg), with a range of -2.37 to -6.21 kg/m^2^, while liraglutide demonstrating a -3.03 kg/m^2^ reduction [4]. The Semaglutide Treatment Effect in People with Obesity (STEP) trials 1-8 have shown that subcutaneous 2.4 mg semaglutide has an average weight loss of up to 16% [12]. This number is important as recent literature has suggested that weight loss from bariatric surgery at around 15% can lead to remission of type 2 diabetes [13-15]. However, the current longest-term trial with semaglutide is two years compared to bariatric surgery which has been evaluated with trials exceeding a decade. Therefore, further research is required to elucidate the long-term weight loss effects of GLP-1 RAs.

The article "Comparative Efficacy of Semaglutide Versus Liraglutide or Efinopegdutide on Weight Loss in Obese Patients: A Systematic Review and Meta-Analysis" was published in 2024. Journal: Cureus.

Both semaglutide and liraglutide have been found to produce dose-dependent weight loss. O'Neil et al. found that a lower dose of semaglutide (0.2 mg) led to greater weight loss than 3 mg of liraglutide. Additionally, at higher doses of semaglutide, continued weight loss after the 52-week trial was observed. At doses of 0.2 mg, 0.3 mg, and 0.4 mg, semaglutide produced significantly more weight loss than liraglutide [4]. Rubino et al. in STEP 8 also found a statistically significant improvement in weight loss with semaglutide compared to liraglutide, with averages of 15.8% and 6.4%, respectively. Greater proportions of weight loss ≥10%, ≥15%, and ≥20% as observed with semaglutide versus liraglutide were 70.9% versus 25.6%, 55.6% versus 12%, and 38.5% versus 6%, respectively [10]. Three included studies utilized 1.0 mg semaglutide as the subsequent 2.4 mg (one study) version was not currently available during the study period.

In mouse models, semaglutide compared to liraglutide has been shown to affect more regions in the hypothalamus, hindbrain, and other neural pathways that were involved with appetite control, reward circuits, and energy expenditure [16]. Thus, semaglutide’s superior weight loss has been theorized to be a result of improved metabolic activity via neurohumoral pathways and decreased compensatory downregulations of energy expenditure [17]. Additionally, recent trials have also found that GLP-1 agonists administered weekly had greater levels of adherence compared to once-daily treatment [18,19].

GLP-1 RAs have also been demonstrated to affect levels of adipokines, which can be classified into pro-inflammatory (leptin, resistin) or anti-inflammatory (ghrelin, adiponectin) molecules. Of these, leptin plays a role in modulating body weight and fat deposition by inhibiting appetite in the hypothalamus [20]. Thus, increased leptin concentrations are correlated with decreased body weight, but elevated levels of leptin can be found with increased body fat levels seen in patients with obesity, suggesting an endogenous resistance to leptin [20]. Resistin plays a regulatory role in insulin resistance and is reported to possibly play an important link between obesity and the development of T2DM [21]. A meta-analysis of RCTs evaluating the effect of GLP-1 RAs found a significant decrease in leptin (WMD: -4.85 ng/mL, 95% CI: -9.32 to -0.38, p=0.03) and resistin (WMD: -1.40 ng/mL, 95% CI: -2.78 to -0.01, p=0.05) [21]. Adiponectin, another adipokine, plays an important role in insulin sensitivity and studies have found that patients with obesity and T2DM have lower levels of this molecule. Increased body fat has been associated with a dysregulation in adipokine levels, thus possibly contributing to obesity-related sequelae [22]. Thus, reductions in weight have been associated with increased adiponectin concentration. A meta-analysis of 20 RCTs after GLP-1 RA usage found a significant increase in adiponectin levels (WMD: 0.59 ug/mL, 95% CI: 0.10-1.08, p=0.02) [22]. GLP-1 RAs also demonstrate other positive changes beyond weight loss and glycemic control. A longitudinal study by Al Refaie et al. found a reduction in visceral fat percentage, LDL cholesterol, and triglycerides, and an increase in adiponectin levels (all p<0.05), indicating a reduction in insulin resistance and inflammation levels [23]. Additionally, these agents have an emerging function as anti-inflammatory agents, as GLP-1 receptors are present in immune cells. These interactions can modulate immune cell signals and suppress the production of pro-inflammatory cytokines such as IL-1B, IL-6, and TNF-α, while promoting the production of anti-inflammatory cytokines such as IL-10 [24].

The article "Comparative Efficacy of Semaglutide Versus Liraglutide or Efinopegdutide on Weight Loss in Obese Patients: A Systematic Review and Meta-Analysis" was published in 2024. Journal: Cureus.

Adverse Events

The most common AEs were mild to moderate gastrointestinal (GI) symptoms such as nausea, vomiting, constipation, and diarrhea [11]. Across the STEP trials, rates of GI symptoms ranged from 10.3% to 82.2%. Discontinuation due to GI AEs was low ranging from 0.8% to 4.5% [18]. In STEP 8, semaglutide and liraglutide had a discontinuation rate of 3.2% and 12.6%, respectively [10]. Uptitration of these drugs is common; therefore, careful monitoring can decrease the risk of these symptoms [11,18]. Similarly, in this study, the most common AEs were also GI symptoms and were transient in duration. Despite the substantial weight loss induced by GLP-1 RAs, long-term adherence is challenging given the substantial cost and GI AEs associated with these agents. Up to half of patients who were initiated on a GLP-1 RA discontinued their treatment after one year, and notable weight regain was observed once treatment was discontinued [25].

Obesity treatment and management is multi-factorial and should ideally be tailored to be personalized for each individual. Age, pre-existing medical conditions, economic status, drug tolerance, and drug interactions will differ greatly between patients. Although GLP-1 RAs have been shown to reduce weight, the effect on overall body composition is unclear in patients with obesity. In type 2 diabetes studies, there has been a trend of decreased lean mass and fat-free mass, although not in a significant manner. Therefore, it is important to keep in mind the effect on body composition rather than strictly the weight loss effect [26-29]. The global economic burden of obesity and subsequent weight loss interventions can not be understated with both medication and bariatric surgery. In 2019, the estimated economic impact of overweight and obesity was 2.19% of the global gross domestic product, with a projected rise to 3.29% by 2060 [30]. A cost analysis of two RCTs of semaglutide and liraglutide found that the cost to produce 1% of weight loss is $1845 and $3256, respectively [31]. Lifestyle interventions coupled with GLP-1 agonist treatment may also provide an even greater weight loss outcome. Several preliminary studies found that liraglutide combined with exercise improved weight loss and maintenance more than liraglutide or exercise alone [3,5]. More recently, it was found that combined liraglutide and exercise also reduced inflammation, cardiometabolic risk, and metabolic syndrome [32,33]. Future studies should involve larger trials directly comparing the effect of different GLP-1 agonists along with the newer drugs that act on more than one receptor such as tirzepatide and retatrutide in both patients with diabetes and/or obesity.

These findings provide valuable insights but highlight significant limitations that warrant attention. First, the current literature regarding weight loss in patients with obesity primarily had comparisons between semaglutide and liraglutide and only one with efinopegdutide. The other currently available GLP-1 agonists that have been used for weight loss are utilized only in patients with type 2 diabetes. Second, 1.0 mg semaglutide was also included, based on studies that conducted their clinical trials before the 2.4 mg version became available. Additionally, both subcutaneous and oral semaglutide were included which may be a confounding factor. Third, two of the included studies were observational cohort studies, and three did not have a control group. Therefore, the study designs make it difficult to sufficiently conclude the superiority of one drug over another. Fourth, three studies included patients with confounding factors as follows: two in which a GLP-1 agonist was administered after bariatric surgery for weight regain, and one in which the patient population had non-alcoholic fatty liver disease. Future studies should include direct comparisons between liraglutide, semaglutide, and tirzepatide, as well as other emerging weight-loss pharmacotherapies, to expand the evidence base. Standardizing dosages (e.g., focusing on semaglutide 2.4 mg) and delivery methods would help address confounding factors. Conducting well-designed randomized controlled trials with homogenous populations and control groups is crucial to establish clearer conclusions. Additionally, exploring these therapies in diverse clinical scenarios would enhance their applicability.

The article "Comparative Efficacy of Semaglutide Versus Liraglutide or Efinopegdutide on Weight Loss in Obese Patients: A Systematic Review and Meta-Analysis" was published in 2024. Journal: Cureus.

## Conclusions

Semaglutide, liraglutide, and efinopegdutide have demonstrated mean reductions in body weight of 12.2 kg, 7.9 kg, and 8.6 kg, respectively, with moderate to high rates albeit low severity AEs. Future studies should prioritize head-to-head comparisons of modern GLP-1 RAs, such as efinopegdutide, tirzepatide, and retatrutide, to assess their multi-receptor effects on weight loss. Additionally, evaluating long-term safety and identifying the most effective regimens will provide critical insights for clinical practice. This will help close the existing gaps in optimizing obesity treatment.
